The article "Animation Narrative on Stress Relief and Psychological Cognitive Development in Adolescents" was retracted in 2023. Reasons: signs of a paper mill; suspected computer-generated content; unreliable results or conclusions; concerns about the data.

# Animation Narrative on Stress Relief and Psychological Cognitive Development in Adolescents

**DOI:** 10.1155/2022/1111488

**Published:** 2022-09-02

**Authors:** Qian Jiang, Li Ma, Min Yue

**Affiliations:** ^1^Art Institute of Xiangtan University, Xiangtan, Hunan 411105, China; ^2^The First People's Hospital of Xiangtan City, Xiangtan, Hunan 411100, China

## Abstract

As the atmosphere of domestic animation is getting stronger and stronger in recent years, its proportion in the process of public aesthetics, entertainment, and consumption is increasing; thus, the relationship between the audience and works has become an important academic focus. The theatrical animation in the animation industry has become the category that needs to be focused on and changed in the development process of domestic animation because of its characteristics of receiving attention from all-age audiences. Because of the diversified audience levels faced by theatrical animation, it is particularly difficult to coordinate the needs of each audience level, coupled with the long-term influence of Japanese and American animation; the trend of pop culture led by network culture; the inheritance, excavation, and reconstruction of national culture; and other cultural environment and creative thinking intertwined, making the construction of the independence of domestic animation appear more and more difficult. The purpose of this paper is to analyze the theoretical study of the healing elements of Natsume Yojimbo and to analyze the creation of Chinese traditional ink and wash in the creation of our own works. It is concluded that the thematic choices are based on two categories: emotions and dreams, which focus on personal life experience and universal concern for human life. The character construction is divided into three aspects: self-resistance and self-reflection, self-vision and self-actualization, and traumatic experience and self-rescue to explain the complexity and diversity of the characters' growth connotation. The narrative perspective constitutes the perspective from which the issues are viewed. The omniscient perspective allows for the coexistence of complex character relationships and a clear storyline, while the limited perspective reveals certain emotional tendencies. The narrative mode presents the moral of the text with cause-and-effect narrative, embellished group narrative, and dreamlike polyphony narrative. Finally, the article discusses the realistic dilemma of the growth narrative of domestic online animation and tries to put forward feasible development suggestions in response to the problems at this stage.

## 1. Introduction

With the rapid development of the global economy and the acceleration of urbanization in recent years, life in big cities has become more stressful and impatience and anxiety have become a common phenomenon [1]. The body and spirit are struggling in the whirlpool of social currents, and the emotions are struggling to survive in the boredom of the crevices, and the body and mind have accumulated a lot of pressure and need healing power to nourish the soul and soothe the heart, just like a traveler in the desert needs water to quench his thirst and save his life [2]. Healing music, healing animation, healing movies, healing pictures, healing animals, are warm things like the spring breeze sprouting young grass on the Buddha's face in spring [3]. In 1999, Ryuichi Sakamoto, the godfather of Japanese music, released the single “BTTB,” which inadvertently achieved a great success as a healing genre and formed a “healing boom” for a period of time. The term “healing” has been used more widely since then [4]. Nowadays, the term is used in many ways, including healing movies, healing comics, healing games, and healing photography [5]. They are mostly used to relax and soothe people, to give constant comfort, to soothe hurts and to give people positive strength [6]. The reasons why the “healing boom” is in full swing in China are similar to the context in which it arose in Japan [7].

After the burst of the bubble economy in Japan, the society began to feel uneasy and tired of overstimulation. Overstimulation is actually a form of masochism, because humans are superior creatures who try to avoid danger and defend themselves, so they begin to seek a cure [8]. This approach has worked to a large extent because a man instinctively knows what he must do. The search for healing is not so much an individual act of different people but rather a necessary need of the times, an activation of the healing capacity of society. Contemporary Chinese society is no longer satisfied with the simple “pleasing to the ears and eyes” but pursues “pleasing to the heart and mind,” not only for the external sensation of the body but also for the inner satisfaction of the spirit [9]. In recent years, comparing Chinese and Japanese culture, we can find that many cultural phenomena in China today originate from Japan, whether it is the “cat economy” or “healing culture,” and the living conditions of young people in contemporary China are becoming more and more similar to those in neighboring countries. It is undeniable that in contemporary China, where anxiety and depression are on the rise, the consumer good category of healing culture has a very broad market prospect [10]. The fast-paced and depressing life of today makes people fatigued, so choosing to watch an animation is a good medicine for relaxation. Most of the "healing" animations are real life themes, full of friendship, emotion, love, brightness, positivity and happiness; there are people laughing a heartwarming fragment, as well as comfort, healing heart wounds, and repair heart defects of the soundtrack and tone. For example, “Natsume Tomodachi,” “Fruit Basket,” and “Honey and Clover” [11].

We can see that although “healing culture” originated in Japan, it has also had a profound impact in China. Currently, domestic “healing” content accounts for a relatively small share of the market and domestic consumers' demand for healing cultural products is increasing rather than decreasing. Therefore, content producers in the cultural industry can create such products to meet the market demand and gain economic benefits, which will also promote the development of China's cultural industry in the direction of industrialization and refinement. For the audience, as the domestic “healing” content joins the competition, the nervous and restless psychological state of social life will be gradually relieved. This is an era when the public needs to be healed, and the birth of domestic “healing” masterpieces is just around the corner. On the other hand, traditional cultural themes of animation works are emerging and the audience also has a high expectation of works with Chinese classical aesthetic style. The relationship between anime culture and ideological and political education is summarized through reading domestic and foreign literature; the various cultural ideas contained in Japanese anime works are analyzed through the text; the reasons why Japanese anime culture is popular among youth and the negative and positive effects of Japanese anime culture on youth groups are summarized and analyzed through questionnaire surveys, and corresponding countermeasures are proposed for the negative effects. “To solve the negative influence of Japanese anime culture on the youth group at source, it is necessary to construct anime cultural works with Chinese characteristics and give full play to the function of Chinese anime culture in thinking and educating people. The article first defines the concept of “network animation.” The author then analyzes the context of the growth narrative of domestic network animation and believes that the Internet itself, the cultural phenomenon of pan-entertainment, and the target audience have influenced the characteristics of the growth narrative. The article then explores the growth narrative characteristics of domestic online animation texts from four aspects: theme selection, character construction, narrative perspective, and narrative mode.

## 2. Related Work

Anime works did not become mainstream culture at the beginning of its existence, so there are few studies on anime culture [12]. In the 1950s, anime culture was studied in the United States but these scholars held an opposing attitude toward anime culture, believing that anime works were associated with the wrong ideology of youth and violent crime cases. With the progress of the times, more and more excellent anime works have emerged and the impression of the academia on anime culture has changed and issues such as anime culture and the ideological and moral cultivation of youths have received more and more attention [13]. Even so, as a subculture, the study of anime culture in academia is only limited to literature, pedagogy, psychology, and communication and the research field is also biased to the study of the anime industry and anime history [14]. The role of animation culture in ideological and political education still needs to be explored and studied by scholars. In the 1960s, foreign scholars generally considered anime culture as “spiritual opium.”

In 1954, Fredric Wertham, an American psychologist, argued that unabashed violence in anime could lead young people to delinquency. In 1954, Fredric Wertham, an American psychologist, argued that unabashed violence in anime could lead young people to delinquency and his most widely known book, Seduction of the Innocent (1954), led directly to a congressional investigation of the comic book industry and the establishment of the Comic Code Authority (CCA), a self-regulatory body for the comic book publishing industry [15]. Since then, all comics have been required to be licensed by the CCA and have the CCA logo on the cover before they can be shipped and sold [16]. By the early 1980s, scholars, led by professor Alex, showed through practice that there was no obvious relationship between the content of anime works and incidents of youth violence. From then on, the academic community began to pay attention to the positive value of anime works. Japanese anime enjoys a certain influence worldwide, and there are more monographs on Japanese anime research, but most of them explore the ideological connotation of anime works and do not explore too much the ideological and political education function of anime culture [17]. In “Partners of Ghibli,” Toshio Suzuki emphasizes the ideological concepts embedded in anime works as the key to attracting audiences: “movies that contain philosophy, ways of being, and inner issues are more likely to sell.”

A review of the history of Japanese anime reveals that anime creators can express their ideas through their anime works, which can have a subtle influence on the thoughts and behaviors of anime audiences [18]. Japanese anime can be divided into four development periods. The first period is the budding period (1917–1945), represented by Kiyotaro Kitayama, Kenzo Masaoka, and Mitsuishi Yorio. In 1944, Kousei Yorio's “Momotaro—The Sea Gods” was suspected of glorifying Japanese militarism. The second period is the exploration period (1946–1973). In 1945, after Japan's defeat, the antiwar animated films were more popular. This period laid the foundation of the undefeated Japanese animation industry, represented by Osamu Tezuka, the “god of Japanese manga.” Osamu Tezuka's red book “Shinboshima” was the prototype of later manga one shots, and in 1961, he founded the Osamu Tezuka Animation Production Department, which sparked a revolution in Japanese animation. In some of his works, Osamu Tezuka launched a sharp criticism of the ills of society that resonated with audiences [19]. The third period is the mature period (1974–1989), represented by the master of animation Hayao Miyazaki. The animated films such as “Valley of the Wind” and “A Thousand and One” are not only beautiful and detailed but also contain various ideas that touch the audience's heart and provoke them to think about themselves, nature, and life. The fourth period is the refinement period (1990–present) [20]. The anime industry has become the mainstay of Japan's economy and enjoys an important position in the world's animation industry. The Japanese government used “anime diplomacy” to successfully reverse the decline after the defeat in World War II and reconstruct the image of Japan in the world. According to Osamu Tezuka's concept of “the age of signs,” Japanese anime has become a sign of communication among teenagers and watching Japanese anime has become one of the daily activities of contemporary teenagers and the hidden ideology in Japanese anime works has a subtle influence on the values of teenagers.

## 3. Constructs of Animated Narratives for Adolescent Stress Relief

### 3.1. Restrictive Narrative Perspective

The essence of film and television art is to tell a story through different images, and the creator presents the story to the audience according to the set perspective. Who tells it and from which perspective it unfolds is the narrative perspective, as shown in Figure 1. Narrative perspective is a concept in the theory of narrative. The narrative perspective of animation works, as the main expression of animation art, is associated with the characteristics of the style and type of animation. “Events, whenever they are described, are always described from a certain ‘visual' range. A point of observation has to be picked, i.e., a certain way of looking at things, a certain perspective.” The narrative point of view in a film or television production consists of the use of the camera, the setting of the characters, the way the story unfolds, and so on. Different narrative perspectives also show the different narrative styles of the creator, which is an important part of the conception of the work. In “Natsume Tomoyo,” the author presents the story to the audience from a limited point of view that is similar to the first-person writing style of a novel. The main character, Natsume, takes on the task of narrating the story, leading us into his fantastical world and experiencing the events that he experience in order to appreciate his feelings. This limited narrative perspective allows the audience's eyes to remain in the character's perception. In the narrative process, the author's attitude is unconsciously preserved and the audience's observation of the character through the first perspective makes the characterization more believable and enhances their identification with the protagonist's worldview and values of life. At the beginning of the work, the viewer is told in the form of an off-screen voice from the protagonist's first perspective. He has been misunderstood because he has been able to see demons since he was a child, and he lost his parents and lived with different relatives until he was adopted by the kind-hearted Fujiwara couple; “I must not give them any trouble. This kind of real feeling of facing the characters can enhance the viewers' sense of identification. It makes the viewer's feeling switch from loneliness to warmth. It makes people feel warm and loving involuntarily.

Compared with social and ethical themes, military themes, and other themes, the daily themes of campus friendship and affection can capture the attention of most audiences. Friendship and affection in school are the experiences of almost everyone in contemporary society, so the themes that closely follow daily life can enter the hearts of viewers. The audience can find their own shadows in the main characters and see their own unpleasant past and frustrations, but they can still stand up and shine in their small lives. Therefore, only works that are full of profound understanding of real life can evoke the aesthetic recognition of the audience. A campus is a place where we all experience not only learning knowledge and acquiring survival skills but also gaining friendships, teacher-student relationships, and even love; where we improve our outlook on life, values, and worldview; and where gain new perceptions of a family. We have our first emotional collision in the rich campus life, encounter unprecedented setbacks, and fight bravely before. Natsume is a Japanese high school student who has the same daily worries as us but has an extraordinary side to him. Since childhood, he has been able to see the demons that others cannot see and the demon spot has become a friend to protect each other and embark on a difficult journey to return the name to the demon. The theme of the story is a fusion of Japanese monster culture into modern school life, which not only brings the audience closer but also attracts young viewers' attention in a novel way. It is thought provoking and evocative and thus calms the anxiety of people.

### 3.2. Linear Narrative Structure

Each episode of “Natsume Yojimbo” is limited to 20–30 minutes. It cannot tell a big story in a short time, but it uses one or two episodes to tell a precise content of returning a name to a monster. From the time that the main character meets the teacher of the monster class and forms a team to return the monster's name, a touching story about the monster is told. Each subsequent episode tells a story of returning the names of the monsters, and there is no juxtaposition between the monsters, so each episode can be read separately without any obvious connection to the next. This short and single story structure will not cause viewers to bother with the drama, and they can watch each episode with a relaxed mind. The single linear narrative with only one main line of plot throughout the story allows the viewer to focus on the main character's thoughts and reflections on the story itself. The story is structured with simple character relationships, and each episode begins and ends with a simple theme: the return of the demon's name by the main character, Natsume. The main character's classmates, friends, and relatives are all relationships that revolve around the main character and do not portray other social attributes or crossover relationships. The simplicity of the character relationships allows the viewer to clearly understand the author's intentions, grasp the character attributes, and help the author portray the characters. Each episode has a different story content, but all of them follow a delicate and introspective emotional line, which constitutes the main line of the whole story, as shown in Figure 2. In modern society, young people like to stay at home more and more; the prevalence of otaku culture and the increasing social pressure make them depressed. The main audiences of animation works are students, teenagers, and newly working adults.

The vivid portrayal of characters is also an important part of healing animation. The characters can reflect the culture of animation, and the characters with personality and infectious power are very outstanding for the works, as shown in Figure 3. The nonrealistic animation characters are the images created by the creator with rich imagination and all the wisdom. Therefore, the characters in animation become the key of an animation, and quality characters are the shape of an IP, which will continue to drive the development of the animation industry chain after the story is over. “The main character is usually at the center of the conflict and is the main actor in the story.” In most of the “healing” animation, the main characters are usually set as ordinary characters. Rarely do they have a prominent personal image of American heroism.

The main character, Takashi Natsume, is a high school student with all sorts of little flaws, a little lazy and a little dumb, and he needs to go to school, which is our own life. This kind of ordinary character setting makes it is easier to approach the audience and create empathy. Although the main character of a healing animation has an incredible experience, he also has daily worries like ordinary people. But the main character with troubles will not fall down but relies on themselves and the strength of the people to overcome difficulties. Natsume, who has been able to see monsters since childhood, has unpleasant memories of human interactions. In Natsume's past memories, he was always the one who was misunderstood and hurt. The monsters always intentionally or unintentionally scare Natsume and even in his side deliberately create some trouble. And these injuries are not only from the demon's fright but also from the disgust of people around. As a child, Natsume always speaks frankly the world in his own eyes. The things that existed in his eyes were invisible to others. Therefore, early in the story, no one on the human side could understand him and he was upset by the fact that he had left the group because of the demons and could not choose the demon side. He can only stand in the middle ground and passively accept what is happening around him. In the real world, there are also many similar bullying phenomena, where you may be bullied for not agreeing with your classmates about certain things or for having excellent abilities. The first-person narrative perspective with a restricted viewpoint determines that the structure of the story should not be too complicated, too complicated story lines will lose the essence of warm and healing animation to give people relaxation, and the up and down episodes looking for character relationship story lines will defeat the viewers' original purpose of enjoying healing animation to release stress and relieve pressure.

In the modern society, human beings are living in a forest made of steel and concrete, working and living in a square box where all we see is the squeeze of living space and the isolation between people. The proud ancient Chinese gardens with their five steps and one view of nature no longer exist and are almost a luxury. The city skyline is blocked by skyscrapers towering in the sky, making it difficult for people in the city to get close to nature. Nature has become a resource that humans convert into profit instead of a source of life that they depend on for survival and emotion, as shown in Figure 4. In this paradox, people seek a healing experience of returning to nature. With this in mind, a healing culture with elements of nature has emerged. In the “healing” animation, Miyazaki's works are almost full of this “nature worship.” The scenes in his animation are almost the benchmark of scene design in the animation industry, and his scene materials come from life but are higher than life. Hayao Miyazaki has always emphasized that man and nature are one, and the metaphorical meaning of most of his works lies in the harmonious relationship between man and nature.

The author, Yuki Midorikawa, says that he grew up in the countryside and has a special affection for nature. It is this interplay of nostalgia and childhood memories that allows the author to create fascinating works with a strong sense of humanity. The real-world scenes of mountains, trees, and shrines that appear in the scenes are treated with the author's personal emotions, thus causing the audience to have a stronger empathy. Natsume, the main character in “Natsume Tomonobu,” lives in a distant relative's house in the countryside and likes to walk in the forest to escape from the people around him. In many scenes, the sunlight spreads through the woods on the earth and we can, like Natsume, calm our hearts through this sunlight and blue sky. As an ordinary high school student, Natsume always wears a white shirt and simple plain clothes, which also reflects the character's plain and simple character to bring the audience closer. Each episode features a lush forest, a colorful summer festival, and a Japanese house with a fish pond. The green color that purifies the heart, the orange color that warms the heart, the pink color that symbolizes love, the blue color that opens up the mood, and the transparent color of the clear pond water are the colors that make up this typical “healing” animation.

### 3.3. Real-World-Based Emotional Expression and Stress Release

Color is the decomposition of light, which plays an important role in regulating the feelings of our life. Color affects people's emotions under the role of human perception and will change with the changes in the living environment in which people live. When analyzing the color performance of a scene, it is inseparable from the artist's personal creative style, as shown in Figure 5. When creating a scene, the artist will blend the style with the emotion of the story and process the real colors to form a more intuitive expression of the emotion and to bring out the atmosphere of the theme. By comparing the color performance of healing animation scenes, we find that most artists will use some similar expressions in creating scenes, mostly in light colors in the scenes that show beautiful healing. In the animation scene, through the image processing of scattered scenes and overexposure, the details of light and shadow enrich the scene, create a fresh and warm visual effect, and make the whole animation give a comfortable experience. Such colors neither give people visual stimulation nor instantly grab the attention of the audience's eyes. According to color psychology, different colors of the set will have an important impact on the audience's psychology. Most fast food restaurants are decorated with warm colors like red and yellow to give people a feeling of excitement and thus promote appetite and speed. Hospitals and libraries, which require quiet places, are mostly decorated with cool colors such as blue and green, which can play a role in calming the mind and stabilizing the emotions. Unlike American commercial animation, which only pursues bright and vivid visual effects and ignores the spiritual aspects, the colors used in Miyazaki's animation represent his profound themes and rich cultural connotations. The shape of the scene set is also based on the real world in the author's mind and artistic creation to draw that this is also a reflection of the artist's living environment and life times.

## 4. Development of Psychological Cognition

The original “healing” culture originated in the field of music. In addition to the lines, the soundtrack is also a very important part of the animation. Good music can make the film and television works more famous, and the music of Hayao Miyazaki's animation works is a typical example of success. Years after the work was shown, the Sky City concert held by Jean Hisaishi is still touring the world. The music has a calmer style and positive lyrics, helping the audience to calm their minds and relieve anxiety. So much so that when you hear the familiar melody and catchy lyrics, you will think of the plot of the animation. The audience's mood will change with the music. Theme songs and interludes are mainly active and animation images with the role of narrative rendering mood and usually have a long-term impact on the audience. According to the contemporary American film theorist Bordwell, “the rhythm, tempo, melody, harmony, and instrumentation of music can influence the audience's emotional response” and the selected repertoire is shown in Figure 6; based on the plot of the animated story, the main ideas are conveyed and the emotions are rendered. In the work for the development of the storyline to do a push, articulation can play a guide role. For the audience, sometimes, the theme music can also be used to capture their hearts and appetites. This allows the audience to enter the story quickly. In animation, although the scene only supports the existence of the characters, it is an indispensable part of the picture. It can be said that the psychological impact of color on the audience is mostly through the drawing of the scene.

With the development of domestic cinema animation, more and more phenomenal animation works have appeared in recent years and its accompanying topicality is that nowadays, the network era cannot be ignored. In order to keep up with the trend, people have to spend time and money to go to the cinema and watch the most popular animation. Whether or not they have seen the most popular films also has a serious impact on social interaction, especially among students and young people. By looking at the changes in microblogging topics before and after the release of “Nezha: Birth of the Demon Child” (see Figure 7), “Nezha” generated a lot of buzz before its release, such as “Is Nezha a boy” and “Nezha and AoBing.” After the release of the film, the topic of “Nezha's head,” “Nezha's pockets,” “AoBing should be called Nezha,” “Why Nezha can't beat Sun Wukong,”, etc. caused a lot of discussion. “Why can't Nezha beat Sun Wukong?” and other topics were hotly debated. Composer Quincy Jones believes that good music and images should be combined in such a way that “the theme music sounds as if it flows naturally from the film's wonderful images.”

In the parent-child activity of leading children to watch movies together, it is especially important whether we can have common topics with children and whether we can bring certain educational significance through watching movies. The creation of some domestic cinema animation nowadays has basically sorted out the relationship between “teaching” and “fun.” At the same time, in recent years, domestic animation has gradually developed from a young audience to an adult audience, making audiences of different ages fall in love with watching animation. It is worth mentioning that in the top ten domestic theatrical animation box office rankings from 2009 to 2019, five of the “Bears” film series are on the list (as shown in Figure 8), which must be seen to be inseparable from the acceptance of adult audiences, in addition to the drive of its original TV animation influence. This shows that the movie has broken through the low-child-oriented mode of its TV animation in terms of production, character design, and storyline, with a comprehensive combination of funny lines and buzzwords and a positive energy blend of justice, responsibility, affection, and friendship, which has been enjoyed by children as well as recognized by adults. Measure the success of a theatrical animation in addition to the box office; another important factor is whether the animation itself has a topic.

Internet culture is a kind of mass culture; people can freely get a lot of information from the Internet, also freely analyze and reorganize according to the information and knowledge that they have, get their own opinions, and have their own views, and at the same time, they are also eager to get some information that can be intriguing to form their own opinions through their own reorganization. With the improvement of the material level of people's life at this stage, people begin to have a deeper understanding of the spiritual world and the main audience of the current cinema animation is growing up with the Internet, from childhood under the influence of American and Japanese animation; the audience of this generation also embodies a significantly different aesthetic psychological characteristics and social and cultural background. Unlike the early domestic animation that advocates truth, goodness, and beauty, people expect to see different views and more complex character settings in the film to satisfy their thirst to show their self-worth shaping, their sense of identity, and their rebellion against traditional elite culture and mainstream culture, as shown in Figure 9. The thread of the story development of “The Great Protector” is a series of things that happen when the Great Protector is looking for the prince of Yiwei who escaped from the palace. In the traditional sense, the prince is an escapist and rebellious person, but from another point of view, we can find that the prince is actually brave to pursue their own goals in life and go forward, without fear of the future, only to achieve self-worth. In fact, he also wanted to realize the value of self-identity in life. This great protector helped the kings of all dynasties to pursue their values. After meeting the needs of children, the adult audience is still paying for the animation film. Then, adults in the viewing space, both as independent viewers but also as children's guardians of the special dual identity, the impact on their cognitive psychology can be an important consideration, while increasing the sense of participation and communication between adults and children is also particularly important.

Omniscient perspective means that the narrator is not a specific character in the film; the film is able to achieve whatever the narrator wants to achieve. The narrator can reach the heart of any character, stay in any hidden corner, and also understand the events that are happening in multiple places at the same time. The audience only needs to be passive in the process of watching the film. The omniscient perspective is the most common narrative approach in domestic network animation, and it is no exception in the growth narrative of network animation. All the storyline development of the film will be clearly laid out in front of the audience, and the audience only needs to receive information easily and constantly and with the development of the story to produce emotional changes, which allows the audience in the current era of universal anxiety to get a moment of relaxation. For example, in the web animation “Fulltime Mage,” the Mu family has always looked down on Mo Fan and wants to humiliate him at the bar mitzvah of his carefully cultivated righteous son. Mo Fan does not know what moves his opponent will make to defeat him, and the Mu family's trickery is presented to the audience by the camera first. In “Dent World,” the main character Jin first arrives in Dent World and meets his best friends Zitang Mirage and Kelly who are adventuring together. The ghost fox Tianchong wants Jin to join the “Ghost Heaven Alliance” and keeps feeding Jin with wrong information. The audience knows the truth before the main character Jin does. The audience knows the truth before the main character Jin that Ghost Fox Tianchong's behavior is actually a trap designed for his own benefit and that he really wants to get the Yuan Power of all people to strengthen himself. The reason for this is that these animation film works find a balance between tradition and innovation based on the premise of modern audience consumption demand and integrate our excellent traditional culture and modern cultural spirit into the animation creation. With the strengthening of China's economic strength and the increase of national self-confidence, the people are more eager to see the excellent culture inherent to their own nation. And the Chinese traditional culture itself is very mature, with a strong infectious force and vitality of culture. There are such traditional virtues such as loyalty, modesty, benevolence, self-improvement, perseverance, impartiality, harmony, hard work, and frugality.

## 5. Conclusion

With the development of network technology and the business model, the development of online video platforms in the new media era is prominent. In order to enhance user stickiness, video platforms are expanding their demand for content, shifting from traditional video broadcasting platforms to independent content production, of which online animation has become an important segment developed by video platforms. The number of online animations has increased dramatically under the good time of developing online animation, and the proportion of domestic online animations with “growth” as the narrative object is remarkable. The article first defines the concept of “online animation.” The author then analyzes the context of the growth narrative of domestic online animation and believes that the Internet itself; the cultural phenomenon of pan-entertainment and the target audience have influenced the characteristics of the growth narrative. Ordinary protagonists from around the setting make the audience feel close. Fantastical events occur, allowing the protagonist to get caught up in the events to attract the audience's attention. Impress the audience with the main character's resilient and warm personality. The characters find their first heart together. The preliminary conclusion of the “healing” animation creation rules will be useful for our animation practitioners to produce animation that is more popular with consumers. Chinese traditional culture has a similar spiritual concept to that of healing culture in its pursuit of natural beauty. The integration of poetic ink elements into the “healing” animation also carries forward and inherits the long history and culture of Chinese classical beauty and highlights the cultural heritage of the ancient civilization. With the wide dissemination of media, the “healing” animation can show its national cultural charm, go to the world and be recognized, and strengthen the cultural soft power of China. This method has a unique reference value for the development of China's animation and game industry. The current stage of domestic animation works began to gradually conform to the modern aesthetic audiovisual habits and spiritual needs of people and in the animation film works into the mainstream values.

## Figures and Tables

**Figure 1:** Animation narrative style.

**Figure 2:** Linear narrative structure.

**Figure 3:** Emotional link between character influence and animation.

**Figure 4:** Summary of natural elements in animation works.

**Figure 5:** Color scenes and emotional expression.

**Figure 6:** Melody and emotion of the theme song.

**Figure 7:** The change of topic popularity before and after the release of the anime.

**Figure 8:** Animation emotional connection and box office relationship.

**Figure 9:** Story source connectivity.

## Data Availability

The data used to support the findings of this study are available from the corresponding author upon request.
